RETRACTED

# Consensus Guidelines for CSF and Blood Biobanking for CNS Biomarker Studies

**DOI:** 10.1155/2011/246412

**Published:** 2011-07-18

**Authors:** Charlotte E. Teunissen, Hayrettin Tumani, Jeffrey L. Bennett, Frode S. Berven, Lou Brundin, Manuel Comabella, Diego Franciotta, Jette L. Federiksen, John O. Fleming, Roberto Furlan, Rogier Q. Hintzen, Steve G. Hughes, Connie R. Jimenez, Michael H. Johnson, Joep Killestein, Eva Krasulova, Jens Kuhle, Maria-Chiara Magnone, Axel Petzold, Cecilia Rajda, Konrad Rejdak, Hollie K. Schmidt, Vincent van Pesch, Emmanuelle Waubant, Christian Wolf, Florian Deisenhammer, Gavin Giovannoni, Bernhard Hemmer

**Affiliations:** ^1^Department of Clinical Chemistry, Neurological Laboratory and Biobank, VU University Medical Center, FdG, P.O. Box 7057, 1007 MB Amsterdam, The Netherlands; ^2^University of Ulm, Ulm 89081, Germany; ^3^Departments of Neurology & Ophthalmology, University of Colorado Denver, Aurora, USA; ^4^Proteomics Unit (PROBE), Department of Biomedicine, University of Bergen, Bergen 5020, Norway; ^5^Division Neurology, Department Clin Neuroscience, Karolinska University Hospital, Stockholm, Sweden; ^6^Neurology, Centre d'Esclerosi Múltiple de Catalunya, CEM-Cat, Unitat de Neuroimmunologia Clínica, Hospital Universitari Vall d'Hebron, Barcelona, Spain; ^7^Laboratory of Neuroimmunology, IRCCS, “C. Mondino Neurological Institute”, Pavia, Italy; ^8^Neurology, Glostrup Hospital, University of Copenhagen, Glostrup 2600, Denmark; ^9^Department of Neurology, University of Wisconsin, Madison 53705, WI, USA; ^10^Clinical Neuroimmunology Unit, Institute of Experimental Neurology, Division of Neuroscience, San Raffaele Scientific Institute, 20132 Milan, Italy; ^11^Neurology, Erasmus MC, Rotterdam, The Netherlands; ^12^Clinical Developement Department, Isis Pharmaceuticals, Carlsbad, California 92024, USA; ^13^OncoProteomics Laboratory, Department of Medical Oncology, VU University Medical Center, 1007 MB Amsterdam, The Netherlands; ^14^Department of Neurology, Leeds Teaching Hospitals NHS Trust, Leeds LS1 3EX, UK; ^15^Department of Neurology and Center of Clinical Neuroscience, 1st Faculty of Medicine and General University Hospital, Charles University, 128 21 Prague, Czech Republic; ^16^Department of Neurology, VU University Medical Center, 1007 MB Amsterdam, The Netherlands; ^17^Neurology and Clinical Neuroimmunology, University Hospital, University of Basel, Basel 4031, Switzerland; ^18^F. Hoffmann- La Roche Pharma, Basel, Switzerland; ^19^Department of Neuroimmunology, UCL Institute of Neurology, Queen Square, wc1n 3bg London, UK; ^20^Department of Neurology, University of Szeged, Szeged, Hungary; ^21^Department of Neurology, Medical University of Lublin, Lublin, Poland; ^22^Department of Experimental Pharmacology, Medical Research Center, Warsaw, MA 02451, Poland; ^23^Accelerated Cure Project for Multiple Sclerosis, Waltham, MA, USA; ^24^Neurology Department UCL, Université Catholique de Louvain, Brussels CA94117, Belgium; ^25^Clinical Development, Lycalis sprl, 1180 Brussels, Belgium; ^26^Clinical Development, UCB Pharma S.A., 6020 Braine l'Alleud, Belgium; ^27^Department of Clinical Neurology, Innsbruck Medical University, Innsbruck E1 2AT, Austria; ^28^Queen Mary University of London, Neuroscience & Trauma Centre, Blizard Institute of Cell and Molecular Science, Barts and The London School of Medicine and Dentistry, London, UK; ^29^Deptartment of Neurology, Klinikum rechts der Isar, Technische Universität, Munich 81245, Germany

RETRACTED

## Abstract

There is a long history of research into body fluid biomarkers in neurodegenerative and neuroinflammatory diseases. However, only a few biomarkers in cerebrospinal fluid (CSF) are being used in clinical practice. Anti-aquaporin-4 antibodies in serum are currently useful for the diagnosis of neuromyelitis optica (NMO), but we could expect novel CSF biomarkers that help define prognosis and response to treatment for this disease. One of the most critical factors in biomarker research is the inadequate powering of studies performed by single centers. Collaboration between investigators is needed to establish large biobanks of well-defined samples. A key issue in collaboration is to establish standardized protocols for biobanking to ensure that the statistical power gained by increasing the numbers of CSF samples is not compromised by pre-analytical factors. Here, consensus guidelines for CSF collection and biobanking are presented, based on the guidelines that have been published by the BioMS-eu network for CSF biomarker research. We focussed on CSF collection procedures, pre-analytical factors and high quality clinical and paraclinical information. Importantly, the biobanking protocols are applicable for CSF biobanks for research targeting any neurological disease.

## 1. Introduction: The Need for Collaborative Biobanking and Biomarker Studies

NMO can be diagnosed based on a blood-derived biomarker, that is antibodies against aquaporin-4, a channel protein present on astrocytes, extensively discussed in other contributions in this special issue. The presence of antibodies against aquaporin-4 has been proven as one of the most successful results of biomarker studies, and is supportive for the idea that central nervous system (CNS) abnormalities are reflected in changes in body fluids. It also proofs the autoimmune component of this disorder and of pathologies that are related to the NMO spectrum disorders, such as longitudinally extensive transverse myelitis. 

RETRACTED

Determination of serum anti-aquaporin-4 antibody levels is a mainstay in the diagnosis of NMO, but the discovery of such disease-specific antibodies is relatively recent [1], and, therefore, further studies in body fluids are warranted. One case report suggested that NMO-immunoglobulin G (IgG), the NMO-associated antibodies that are reactive to cerebellar tissue [1], can be absent in serum, but present in CSF [2]. However, another study on a relative large cohort of patients showed that testing CSF does not increase diagnostic sensitivity [3]. Another recently identified candidate biomarker for NMO is glial fibrillary acid protein (GFAP). Takano and colleagues observed that the analysis of CSF glial fibrillary acid protein is useful in the differential diagnosis between NMO and multiple sclerosis or acute demyelinating encephalomyelitis, and that its CSF levels at disease onset correlated with expanded disability score scale (EDSS) in NMO [4]. However, studies on larger cohorts are needed before drawing definite conclusions. Taken together, no biomarkers are available yet for prognosis or therapy response in NMO and in NMO-related disorders. Therefore, biomarker studies on CSF are ongoing. 

One important flaw in several previously performed biomarker studies in CNS diseases has been the lack of large cohorts to sufficiently power the study. This is especially an issue for such a rare disease as NMO, where a single center will not be able to collect a large cohort within a reasonable time frame. The need for collaboration was the reason for biomarker researchers in Multiple Sclerosis to start a network (BioMS-eu, http://www.bioms.eu/). The aim of this collaboration is to obtain well-proven, high-quality biomarkers, which will be achieved by sharing patient samples, standardization, and improvement of procedures important in the research area. One of the most urgent prerequisites for collaboration was felt to be standardization of biobanking protocols. Therefore, a consensus-meeting was organised and the result was collection and biobanking guidelines, which the network developed and published in 2009 [5]. There are currently major efforts worldwide to professionalize biobanks and the collection and biobanking guidelines established by consensus among 26 groups participating in BioMS-eu (http://www.bioms.eu/) is a major achievement in the CNS biomarker field [5]. One year after publication of the guidelines, over 90% of the BioMS-eu laboratories had already adapted their procedures in agreement with the guidelines. A great use of the guidelines is the applicability for any neurological disease, including NMO, and that it provides guidelines for setting up a novel biobank. Furthermore, it will greatly facilitate biomarker studies in the CNS biomarker research area. In the concensus discussions, we have sought a balance between practicality and scientific rationale, and the background of each decision is provided. Before the consensus, it was clear that large differences were present between collection protocols, highlighting the need to address these differences (Figure 1 and Table 1). In the current paper, we include only the items and their rationale from the original paper that are relevant for biobanking for NMO. Other modifications from the original protocol is an adaptation of item 1 (samples should be pooled if multiple collection tubes are used for one patient), and the inclusion of an item addressing transportation (item 20) and information of some more physiological confounders (item 25). 

RETRACTED

We would like to stress that researchers adhere to these protocols for optimal collaboration in the field of CSF biomarker research. We suggest using Tables 2 and 3 as a checklist for CSF biomarker research and recommend that future studies of CSF biomarker take these issues into account. In discovery-based biomarker research, all these items should be considered carefully before initiating a study. Some procedures may not be possible in everyday clinical practice (e.g., processing within one hour), but less stringent requirements will suffice for specific research questions. Therefore, careful documentation of these issues is crucial to facilitate retrieval of appropriate samples dictated by specific study aims. As indicated before, the procedures for withdrawal and storage of CSF (Table 2) are broadly applicable for any neurological disease. 

Besides methodological issues, ethical approval is a crucial prerequisite for collaboration between international or national centers. The signed informed consent should include a statement that exchange of samples between (international) centers is allowed. Furthermore, to bring a biomarker to clinical practice, one may need patents and the involvement of industrial partners could be needed, who have the infrastructure for large-scale production, quality control procedures, and to reach as many laboratories as possible. For large-scale validation studies, patient samples are of course also needed, and it will be wise to consider this possibility at the start of biobank formation and, if ethical laws permit and the option is perceived to be important, indicate the possibility for industrial cooperation in the patient information and consent.

RETRACTED

Lastly, researchers should be willing to share their samples and information for the benefit of the whole, that is, obtaining reliable biomarkers that can be used for patient care and cure.

## 2. Guidelines for CSF Biobanking for Biomarker Research, Rationale, and Details

### 2.1. Procedure of CSF Collection (Table 2)

**(A) Collection Procedures:**

**Item 1 Volume of Withdrawal of at Least 12 mL**

The CSF volume taken can influence the concentration of biomarkers. Most molecules and cell numbers have a rostrocaudal concentration gradient [6, 7]. If a small volume is taken, the CSF will reflect the composition of the lumbar dural sac, whereas large volumes may reflect the rostral spinal or even ventricular CSF. Therefore, if biomarker concentrations in a sample from a puncture of 2 mL are compared to that in a puncture of 15 mL, this can lead to erroneous results. Also collecting different portions of the CSF for biobanking (e.g., initial and final volumes of the puncture) may introduce errors. Thus, a standard volume of CSF should be collected during lumbar puncture, the first 2 mL can be used for basic CSF analysis (item 26), and the remainder of the sample should be pooled before spinning and aliquoting. At least, the procedure must be recorded. The volume of collected CSF does not correlate with the risk of postlumbar puncture headache [8, 9].

**Item 2 Location of Puncture: Vertebral Body L3–L5**

Usually, diagnostic CSF is obtained by lumbar puncture. Because of the increasing gradient in protein concentration from ventricular to lumbar CSF [10], the site of CSF withdrawal must be recorded. When CSF is taken from other locations such as the cervical cisterns or from the lateral ventricles (e.g., ventricular drainage), this should be documented.

**Item 3 Removal of Bloody CSF Samples**

A traumatic tap causing blood contamination of CSF occurs in about 14–20% of standard lumbar punctures [11]. For biomarkers that have high serum concentrations, such as coagulation factors, blood contamination can lead to false positive results. In addition, blood proteins lead to suppressed matrix-assisted laser desorption/ionization-mass spectrometry (MALDI-TOF/MS) proteomics patterns in CSF. This suppression by blood proteins is, however, highly reduced after removal of the blood cells by centrifugation prior to initial freezing [12, 13]. Recording of erythrocyte count is essential to select CSF samples appropriate for these measurements. CSF samples with an erythrocyte count above 500/*μ*L should not be used for biomarker studies.

**Item 4 Use of Atraumatic Needle (Sprotte or Whitacre Needle)**

There is no evidence that the type of lumbar puncture needle influences biomarker concentrations. However, atraumatic needles are best tolerated by patients, and are associated with a lower risk for postlumbar puncture headache, that is about 12% for a needle size of 20–22 G compared to about 70% for a needle size of 16–19 G [14, 15].

RETRACTED

**Item 5 Use of Polypropylene Collection Tubes**

There are several reports showing that the type of collection tube influences biomarker outcomes, for example, total tau proteins and amyloid *β* peptides [16]. Therefore, standardization is important. We propose to use polypropylene tubes, with their low protein binding potential, for collecting CSF. No additives should be used. Glass tubes should be avoided, due to safety reasons for personnel. When multiple tubes are used, the total volume should be mixed after centrifugation to avoid gradient effects.

**Item 6 Time of the Day of Withdrawal**

For biomarkers that are influenced by circadian rhythm, time of withdrawal is important [17]. Since it is often difficult to accomplish standardization of withdrawal time in everyday clinical practice, documentation is necessary to select the appropriate samples to minimize the effect of this variable.

**Items 7 and 8 Serum, Plasma, and DNA Linked to the CSF Sample**

It is important to collect matched serum and/or plasma samples for evaluation of CSF biomarkers because the concentration of the marker in blood often influences that in CSF [18]. Further, serum/plasma pairs are essential to study the intrathecal origin of a biomarker and its CNS specificity. Furthermore, the presence of CNS markers in serum/plasma may aid in disease monitoring. Vacuum tubes that use EDTA (in dried format) are preferred over those that use citrate (in solution) because if tubes containing a standard volume of citrate are filled incompletely, the final biomarker concentration is diluted unequally compared to other samples. Depending on the type of biomarkers and methods of study, we recommend collecting both serum and plasma [19]; for some methods, plasma is preferred over serum and vice versa. Serum/plasma samples should not be haemolysed. We advise to perform a blood draw using vacuum systems, since tourniquet use is related to additional confounding factors in the preanalytic phase include tourniquet time and posture [20]. Furthermore, instructions of the supplier should be followed, such as mixing.

Lastly, DNA collection expands the possibilities for studying the phenotypes and genotypes within individuals. A protocol for storage and handling of DNA can be found in the supplementary files (E-Appendix  1).

**(B) Processing for Storage:**

**Item 9 Storage at Room Temperature Until Spinning and Aliquoting**

For CSF, there are no data available yet that support a preference for leaving the samples at room temperature or at 4°C until processing. For serum/plasma preprocessing temperature is more crucial. To avoid platelet activation [21], serum/plasma samples should be kept at room temperature before centrifugation. Therefore, processing at room temperature for both serum/plasma and CSF, including during and after spinning, is suitable for most studies. Relatively few systematic studies have been performed on this issue. We would recommend exploratory studies to define the effect of temperature on specific biomarkers.

RETRACTED

**Item 10 Standardized Spinning Conditions**

We propose to adhere to a standardized spinning protocol of 400 g for 10 minutes at room temperature when fragile cells need to be preserved for RNA of cell isolation, and otherwise at 2,000 g. For serum/plasma, we propose to spin at 2,000 g for 10 min at room temperature. Standardization of spinning temperature and speed may be important for some biomarkers, although no studies have addressed these specific preanalytical variables for CSF. For plasma and serum, temperature of processing is known to be critical for specific biomarkers [22]. After centrifugation, the supernatant must be aliquoted and stored immediately. If this is not done, the processing time should be documented.

**Item 11 Standardization of Time-Delay between Withdrawal, Spinning, and Freezing**

Studies of the effects of preanalytical variables by MALDI-TOF/MS proteomics (proteins/peptides <20 kD) have shown that the time between sampling and storage is more crucial for specific serum proteins or peptides than for CSF, [12, 13, 23]. For CSF, it was observed that processing within two hours does not lead to artefactual results [12, 13]. For serum, it was observed that small differences in processing time (~10–30 min) can result in changes in the protein profile [19]. Some biomarkers, such as antibodies or specific cytokines, are not very sensitive to sampling and storage conditions [24]. For practical reasons, and in view of the standard of 30–60 min clotting time for serum, we recommend a time delay of 1.5 hours (±30 min) for both matrices. When CSF cells are to be preserved, processing as soon as possible is to be advised as cell numbers decrease quickly. However, in most of the centers, processing of the body fluid samples within one hour is not common practice. Therefore, documentation of time of withdrawal and storage is required in order to select uniform samples. For newly discovered biomarkers, these preanalytical variables should be evaluated.

**Item 12 Use of Small Polypropylene Tubes for Aliquoting**

Due to the same rationale as for CSF withdrawal (item 5), we recommend that polypropylene tubes should be used for aliquoting and storage. Furthermore, vials with screw caps should be used for a secure sealing. The proposed tube size is 0.25, 0.5, and 1 mL.

RETRACTED

**Item 13 Aliquoting**

Freeze/thaw cycles can influence biomarker concentrations [25]. For example, one-time freezing of CSF samples can lead to a highly significant loss of amyloid *β*(1-42) which is decreased a further 20% after three more thawing cycles [26, 27]. By contrast, no effects on CSF proteome profiles obtained by MALDI-TOF/MS have been observed after up to four freeze/thaw cycles [13].

In principle, repeated freeze/thawing of samples should be avoided, as data addressing this topic are available for only a few biomarkers and the response to freeze/thaw cycles of new biomarkers is not known. Thus, splitting the pooled sample in multiple small aliquots is optimal, and possible freeze/thaw cycles should be recorded.

**Item 14 Volumes of Aliquots of 0.2, 0.5, and 1 mL**

Small aliquot volumes are optimal to avoid freeze/thawing and to avoid waste of CSF. Tubes should be filled up to 75% to prevent freeze-drying within the tube, which will affect the concentration of biomarkers, although it may only be a problem if the seal of the cryogenic tubes are not airtight. This issue has not been formally studied and is not referred to in related standard operating procedures [28].

**Item 15 Coding and Use of Freezing-Proof Labels**

Unique codes are necessary to track samples and pair with clinical data. Ideally barcodes should be used to facilitate searching, to aid in blinding the analysis, and to protect the privacy of patients. It is important to have center-unique codes, to track data retrospectively. Labels must be water and frost (−80°C) resistant.

**(C) Storage and Administration of Samples (Table 2, Lower Part):**

**Item 16 Freezing Temperature of −80°C**

Proteins may not be stable at −20°C for years. In one study, the effect of storing CSF at −20°C and −80°C on cystatin C, an abundant CSF protein, was investigated. Cleavage of this protein occurred in all samples stored at −20°C but not in samples stored at −80°C [29]. Apart from the cystatin C truncation, changes in the low molecular weight polypeptide profile due to CSF sample storage at −20°C for three months appeared to be minimal [12, 13]. Oligoclonal bands in CSF may be recovered after several years of storage at −20°C indicating a high stability of immunoglobulins. Nevertheless, self-defrosting freezers must not be used. No data are available showing the benefit of storage of CSF or serum in liquid nitrogen. As this is expensive and not practical for CSF biobanking, there is no basis yet to recommend storage in liquid nitrogen.

RETRACTED

Taken together, we recommend that samples are stored at −80°C to ensure long-term stability of biomarkers.

**Item 17 Location of Samples**

To enable easy tracking and fast relocation of samples, storage information should include freezer location, freezer identification, and sample location within freezer.

**Items 18 and 19: Surveillance of Freezers and Splitting of Samples**

Freezers should be alarm controlled and a sample rescue plan established and documented. All freezers must be registered in a freezer log file. Ideally, daily temperature logs should be available for all freezers. Aliquots of samples should be distributed among different freezers, although not absolutely needed if good surveillance is in place. An empty, an empty back-up freezer should be available.

**Item 20: Transport Conditions and Thawing before Use**

Transport of frozen samples should always be performed on dry-ice, and the volume should be sufficient for transport for minimal 3 days. Preferably, transports are initiated on Monday for the samples to arrive within the same week. Once the samples have arrived and are ready for experiments, excessive thawing temperatures (such as 37°C) are to be avoided to prevent protein degradation. Furthermore, inadequate agitation can cause salt and protein gradients to form in thawed samples.

**(D) Patient Information Requirement in Database:**

**Items 21-22 Basic Demographics, such as Age and Gender**

Information on the age at sampling is needed to allow comparability to age-matched reference values, since many proteins show age-dependent changes, for example, albumin or IgG [30]. Ideally, date of birth and date of sampling are recorded. Gender has to be provided due to variability of markers influenced by hormones.

**Item 23 Ethnicity**

Reference ranges of biomarkers can be influenced by the genetic status [31]. For example, a recent study observed a higher IgG index in African Americans than in Caucasians, unrelated to socioeconomic status [32]. Criteria for race and ethnicity are available via the website of the National Institutes of Health [33].

**Item 24 Treatment at Sampling and Year before Sampling**

It is well known that commonly used drugs for treatment of MS, including immunomodulatory agents and use of methylprednisolone for treatment or prevention of relapses, have an influence on expression of biomarkers [34, 35]. Other treatments could likewise influence biomarker results in NMO patients. Therefore, type and duration of treatment should be documented in detail, preferably beginning at least one year before CSF collection.

RETRACTED

**Item 25 Fasting, Infections and Pregnancies**

Other relevant physiological variables that can influence CSF and blood analyte levels should be recorded including fasting versus non fasting, pregnancy, and underlying nonneurological conditions such as infections [20].

**Item 26 Basic CSF Analysis (Protein, Cell Counts, Erythrocytes, Etc…)**

To enable stratification of patients according to their CSF findings and to evaluate suitability of samples for further analysis, results of basic CSF analysis should be recorded. Primarily, the CSF profile serves for exclusion of other diseases. In addition, quantitative changes of immunological markers are likely to occur depending on disease stage, relapse activity, and medication. Inflammatory processes may influence the blood-CSF barrier function and thereby biomarker concentrations [18].

The presence of Oligoclonal IgG bands (OGB) in NMO is quite distinct from that in MS in that OGBs in MS are persistent, while they are transient in NMO [36, 37]. For example, OGBs were detected in 399 of 411 MS patients (97%) and never disappeared. In NMO, OGBs were detected in three of 11 patients (27%) and always disappeared. The sensitivity of oligoclonal IgG bands is strongly dependent on the method used. We strongly recommend isoelectric focusing followed by immunoblotting and staining for IgG [38, 39]. Preferably, the methods of all routine diagnostic procedures, including oligoclonal banding, should be documented.

**Item 27 Data in the CSF Database in English**

The mask on the database screen could be in the local language, but the underlying files will need to be in English. It is strongly suggested to use a commercially available program, if not a common database for networks like BioMS-eu. The database should also adhere to standardized international units.

## 3. Concluding Remarks

The lists provided in Table 2 can be used as an easy checklist for CSF biobanking for any CNS disease, applicable during setup of the procedures and also as a checklist for recording sample characteristics. It is expected that these standardizations will pave the way for large biomarker studies and fruitful collaborations. In the original paper, we present guidelines for outcome measures to be included for MS biomarker studies [5]. For NMO, standardisation of outcome measures is still needed. Ultimately, these endeavors are to arrive at validated biomarker assays for diagnosis, prognosis, and treatment of CNS diseases and a potential to elucidate relevant disease mechanisms.

## Figures and Tables

**Figure 1:** Results of inventory of collection procedures among 14 European centers with CSF biobanks for MS research in 2006. (a) Other body fluids that are collected simultaneously with CSF. Filled area indicates “yes”; open areas: not collected. (b) Storage temperature of CSF and serum. Open area: −80; closed area: −20; grey area: not collected. (c) Average volume of CSF that is collected per patient per CSF withdrawal. Bars indicate the average and ranges of volume per center. (d) Time-delay between CSF withdrawal, spinning and storage into the freezer. Bars indicate the average and ranges of time per center.

RETRACTED

**Table 1:** Results of inventory on collection protocols among 14 MS Biomarker Research Centers.

Procedure of CSF withdrawal	Previous status among European CSF centers
Type of needle:	71% atraumatic, 21% traumatic, 8% both
Time of the day of withdrawal (important for markers that are sensitive for circadian rhythm)	71% no specific day/time of withdrawal, 29% in the afternoon only
Temperature until storage	57% room temperature, 43% at 4°C
Type of tube:	50% Sarstedt, 29% Eppendorf, 21% other
aliquoting:	Range from 0.2 mL to 2 mL
(1) surveillance of freezers	Present at 93% of the centers
(2) several freezers to split the samples (backup)	Present at 14% of the centers

**Table 2:** Guidelines for procedure of CSF withdrawal.

Item no.	Procedure	Ideal situation
*(A) Collection procedures*		
(1)	Preferred volume	At least 12 mL. First 1-2 mL for basic CSF assessment (item 26). Last 10 mL for biobanking. Record volume taken and fraction used for biobanking, if applicable.
(2)	Location	Vertebral body L3–L5
(3)	If bloody	Do not process further.
		Criteria for bloody: more than 500 red blood cells/*μ*L.
		Record number of blood cells in diagnostic samples.
(4)	Type of needle	Atraumatic
(5)	Type of collection tube	Polypropylene tubes, screw cap, volume >10 mL.
(6)	Time of day of withdrawal and storage	Preferably standardized within each center allowing for intercenter differences in local logistics.
		Record date and time of collection.
(7)	Other body fluids that should be collected simultaneously	Serum
(8)	Other body fluids that should be collected simultaneously	Plasma: EDTA (preferred over citrate).

*(B) Processing for storage*		
(9)	Storage temperature until freezing	Room temperature before, during, and after spinning.
(10)	Spinning conditions	Serum: 2,000 g, 10 min at room temperature.
		CSF: 400 g, 10 min at room temperature/2,000 g if no cells are to be preserved.
(11)	Time delay between withdrawal and spinning and freezing	Optimal for CSF: 1-2 hours
		Optimal for serum: 30–60 min.
		Thus doing “*both body fluids simultaneously*”: ideally within one hour.
		After spinning, samples must be aliquoted and frozen immediately for storage at −80*º*C.
(12)	Type of tube for aliquoting	Small polypropylene tubes (1 to 2 mL) with screw caps. Record manufacturer.
(13)	Aliquoting	A minimum of two aliquots is recommended. The advised research sample volume of 10 mL should be enough for >10 aliquots.
(14)	Volume of aliquots	Minimum 0.1 mL. Depending on total volume of tube: 0.2, 0.5, and 1 mL. Preferably, the tubes are filled up to 75%.
(15)	Coding	Unique codes. Freezing-proof labels. Ideally barcodes to facilitate searching, to aid in blinding the analysis and to protect the privacy of patients.

*(C) Storage conditions and administration*		
(16)	Freezing temperature	−80*º*C
(17)	Additional items on sample collection protocols that must be recorded	Location of samples
(18)	Additional items on sample collection protocols that must be recorded	Surveillance of freezers
(19)	Additional items on sample collection protocols that must be recorded	Splitting of samples over two or more freezers
(20)	Transport conditions	Always on dry-ice, sufficient volume of dry-ice for minimal 3 days of transport.
		Initiated on Mondays.
		Avoid high temperatures for thawing and mix thoroughly.

RETRACTED

**Table 3:** Guidelines for patient information requirement in databases of MS patients.

Item no.	(D) Patient information requirement in databases
	(a) Basic demographics
(21)	(1) date of birth (age if date of birth is not available)
(22)	(2) Gender
(23)	(3) Ethnicity
(24)	(4) Use of drugs, at sampling and year before sampling.
(25)	(5) Actual nonneuronal infections, fasting or nonfasting, pregnancy.
(26)	(6) Basic CSF analysis (CSF cell count, differential cytology, erythrocyte count, oligoclonal IgG bands (which is at least two bands by definition), albumin ratio, total protein (if albumin is not measured), and IgG index)
	(7) Record the methods of routine analysis
(27)	(8) The data in the CSF database should be in English and use Standardized International Units
